# MCU Inhibitor Ruthenium Red Alleviates the Osteoclastogenesis and Ovariectomized Osteoporosis via Suppressing RANKL-Induced ROS Production and NFATc1 Activation through P38 MAPK Signaling Pathway

**DOI:** 10.1155/2022/7727006

**Published:** 2022-09-13

**Authors:** Yuxin Wang, Xiang Li, Shengji Zhou, Jiarui Li, Yi Zhu, Quan Wang, Fengchao Zhao

**Affiliations:** ^1^Department of Orthopaedic Surgery, The First Affiliated Hospital, Zhejiang University School of Medicine, Hangzhou 310003, China; ^2^Department of Neurology, Ningbo Medical Center Lihuili Hospital, Ningbo 315000, China

## Abstract

Osteoporosis is a disorder of bone metabolism that is extremely common in elderly patients as well as in postmenopausal women. The main manifestation is that the bone resorption capacity is greater than the bone formation capacity, which eventually leads to a decrease in bone mass, increasing the risk of fracture. There is growing evidence that inhibiting osteoclast formation and resorption ability can be effective in treating and preventing the occurrence of osteoporosis. Our study is the first time to explore the role of the mitochondrial calcium uniporter (MCU) and its inhibitor ruthenium red (RR) in bone metabolism, clarifying the specific mechanism by which it inhibits osteoclast formation in vitro and plays a therapeutic role in osteoporosis in vivo. We verified the suppressive effects of RR on the receptor activator of nuclear factor-*κ*B ligand (RANKL-)-induced differentiation and bone resorption function of osteoclasts in vitro. The reactive oxygen species (ROS) production stimulated by RANKL and the expression level of P38 MAPK/NFATc1 were also found to be inhibited by RR. Moreover, the promotion of RR on osteogenesis differentiation was investigated by alkaline phosphatase (ALP) and alizarin red S (ARS) staining and the detection of osteogenesis-specific gene expression levels by quantitative polymerase chain reaction (qPCR) and western blotting. Moreover, in ovariectomy (OVX-)-induced osteoporosis models, RR can downregulate the expression and function of the MCU, relieving bone loss and promoting osteogenesis to present a therapeutic effect on osteoporosis. This new finding will provide an important direction for the study of RR and MCU in the study of bone metabolism therapy targets.

## 1. Introduction

Osteoporosis is a disease of bone metabolism, manifested by a decrease in bone density and fragile bones, which can easily lead to fractures. Fractures resulting from osteoporosis are a major cause of morbidity and mortality [1]. Bone metabolism is a dynamic processing in which osteoclast-mediated bone resorption and osteoblast-mediated bone mineralization are two important factors in maintaining its balance. Abnormally activated osteoclast differentiation and increased bone resorption due to osteopenia are one of the important causes of osteoporosis [2]. It is estimated that the prevalence of osteoporotic women over 50 years of age is 32.1%, which is much higher than that of men of the same age by 6%, while the prevalence of women over 65 years of age is 51.6% by 2050 [3]. With the increasing incidence of osteoporotic fractures, which has seriously endangered the quality of life of the elderly population, it is important to elucidate the specific mechanisms that regulate osteoclast differentiation and function to provide new direction and therapeutic targets for the treatment of osteoporosis.

It has been well known that osteoclasts are differentiated from bone marrow-derived monocytes (BMMs) and are the only cells in the human body with bone resorption function [4]. Monocytic precursors gradually fused into multinucleated osteoclasts, which stimulated by RANKL and macrophage colony-stimulating factor (MCSF). In the physiological state, osteoblasts can produce the majorities of RANKL, binding to the receptor activator of nuclear factor-*κ*B (RANK) on osteoclast precursor cells and promotes osteoclast differentiation. It was reported that estrogen promotes the expression of osteoprotegerin (OPG) by acting on estrogen receptors, which competitively bind to RANK and then inhibits mature osteoclast production. This competitive inhibition was supposed to be the substantial mechanism that maintained the balance of bone metabolism through the OPG-RANKL-RANK axis [5]. After menopause, decreased estrogen levels lead to abnormal osteoclast activity. RANKL binds to the RANK on the surface of the cell membrane by acetylation or phosphorylation of the recruitment protein tumor necrosis factor receptor-associated factor 6 (TRAF6) and a variety of inflammatory factors, thereby activating downstream signaling pathways, including phosphoinositide 3-kinase (PI3K)/serine-threonine protein kinase (Akt), mitogen-activated protein kinases (MAPKs), and nuclear factor-kB (NF-*κ*B). Eventually, the activation of NFATc1 is upregulated, a key transcription factor for osteoclast gene expression, which promotes osteoclastogenesis, enhances bone resorption, and causes bone mass reduction [6–8]. In addition, a large number of ROS are produced during the differentiation of osteoclasts induced by RANKL. It has been reported that ROS can further activate downstream MAPKs and NF-*κ*B osteoclast signaling pathways and is closely associated with inducing osteoblast apoptosis [9].

It has been proved that MCU is localized on the inner-mitochondrial membrane, and its protein consists of 351 amino acid residues with molecular weight of about 40 kDa. In recent years, cryogenic electron microscopy (cryo-EM) was applied by researchers to further reveal the precise architecture of MCU. The overall structure of the MCU comprises central pore-forming channel, two coiled coils domain (CCD), and an N-terminal domain (NTD). In addition, it has been found that the pore-forming domain of MCU possesses four identical subunits that composed of two transmembrane helices (TM1 and TM2), respectively. A short stretch of amino acids containing DIME (Asp-Ile-Met-Glu) motif was situated between the two TMs to form a linker [10, 11]. MCU transports cytoplastic calcium (cCa^2+^) into the mitochondrial matrix in an electrochemical gradient dependent, a process that does not rely on ATP hydrolysis for energy and is not accompanied by co-transport of other ions or molecules. The homeostasis of mitochondrial calcium concentration is of great significance for a variety of cellular reactions mediated by intracellular calcium. On one hand, it can effectively regulate the signaling pathways and calcium oscillations in the cytoplasm. On the other hand, it has important regulatory functions for the material and energy metabolism, cell division and differentiation, and cell apoptosis and necrosis within the mitochondria. Besides, the dehydrogenases involved in tricarboxylic acid (TCA) cycle and complexes I, III, IV, and V in OXPHOS are sensitive to mitochondrial calcium (mCa^2+^), which were closely related to the production of ROS [12, 13]. Previous research reports have proved that MCU has a tight connection with inflammatory response, hypoxia injury, tumor cell proliferation, and fat metabolism. MCU expression is upregulated in cancerous tissue, which strengthens calcium absorption in mitochondria and promotes the growth of cancerous tissue both in vivo and in vitro experiments. At the same time, the level of ROS in tumor cells was found to increase with high MCU expression [14–17]. Findings in mice models of ischemic reperfusion injury and hypoxia reoxygenation show that the MCU expression levels elevated during ischemia-reperfusion with a massive mROS generated when blood reentered, causing acute myocardial injury [18]. The Tomar et al. [19] also found that the mice, applied with CRISPR/Cas9 technology to knockout MCU, could sharply inhibit the absorption of calcium ions in mitochondria and delayed the clearance of calcium in cytoplasm, thus reducing the level of intracellular oxidative phosphorylation. Fatty acid accumulation in liver cells also decreased with oxidative phosphorylation levels, revealing the association between MCU and metabolic diseases [20], whereas there has been no research that explores the influence in osteoporosis, which is closely related to the inflammatory response and intracellular calcium concentrations. Therefore, we speculate that MCU could have an important impact on the process of osteoclastogenesis.

RR is a polycationic dye with a linear structure consisting of three ruthenium atoms with a net valence of 6 [21]. It is reported to be the inhibitors of mitochondrial calcium unidirectional transporters, which has an appearance of red crystal that was first used in 1890 for the dyeing of specific fruit acids, gums, and colloids [22, 23]. Later, it was gradually studied in depth in a variety of specific intracellular mechanisms as a drug and found to be a voltage-sensitive calcium channel inhibitor [24]. According to the present researches, RR has significant therapeutic effects on neuronal apoptosis, necrosis, and cardiomyocyte ischemia-reperfusion injury by inhibiting the function and expression of MCU [25, 26]. However, the use of RR to treat osteoporosis by inhibiting MCU has not been reported in the literature. Therefore, in our research, we will reveal the effect of the MCU inhibitor RR on osteoclast differentiation, bone resorption capacity, ROS production, and its specific mechanisms, elucidating its therapeutic effect in animal models of osteoporosis induced by OVX.

## 2. Materials and Methods

### 2.1. Reagents

The alpha modification of Eagle's medium (a-MEM, Lot#12561056), penicillin/streptomycin, and fetal bovine serum (FBS, Lot#10099141) were purchased from Gibco-BRL (Gaithersburg, MD, USA). The cell counting kit (CCK-8) was obtained from Dojindo Molecular Technology (Kumamoto, Japan). Recombinant mouse M-CSF and mouse RANKL were obtained from R&D (Minneapolis, MN, USA), and RR (Cat#1439) was purchased from Tocris Bioscience (Minneapolis, MN, USA) and diluted in PBS. Specific antibodies against P65, ERK (extracellular signal-regulated kinase), JNK (c-Jun N-terminal kinase), p38, phosphor-P65, phospho-ERK (Tr202/Tyr204), phospho-JNK (Tr183/Tyr185), phospho-p38, c-Fos, NFATc1, CTSK, ACP5, Runx2, collagen 1*α* (Col1*α*), GAPDH, and *β*-tubulin were all obtained from Cell Signaling Technology (Danvers, MA, USA). Antibody against MCU (Lot#CL3576) was purchased from Abcam (Cambridge, MA, USA). The TRAP staining kit and all other reagents were purchased from Sigma-Aldrich (St. Louis, MO, USA) unless otherwise stated.

### 2.2. Mouse Bone Marrow–Derived Macrophages (BMMs) Preparation and Osteoclast Differentiation

Primary BMMs were isolated from the femoral and tibial bone marrow of female 8-week-old C57BL/6 J mice. The mice were performed cervical dislocation and then immersed in 75% ethanol for 5 min. The femur and tibia were isolated after removing attached muscle. Subsequently, the bone marrow was flushed out into a 10-cm culture dish with *α*-MEM medium containing 25 ng/ml M-CSF, and the cells were incubated in a 37°C, 5% CO_2_ incubator. The medium was replaced after cultivation of 48 hours until 90% confluence reached. The BMMS were further planted into a 96-well plate at the density of 6 × 10^3^/well with the presence or absence of 25 ng/ml M-CSF, 50 ng/ml RANKL, and different concentrations of RR (0.375, 0.75, and 1.5 *μ*M) to induce osteoclastogenesis. After stimulation for 5-7 days, multinucleated osteoclasts were immediately washed with phosphate-buffered saline (PBS) for three times, then fixed with 4% paraformaldehyde for 20 mins at room temperature (RT), and performed tartrate-resistant acid phosphatase (TRAP) staining for 30 mins.

### 2.3. Differentiation of Osteoblastic Stromal Cells

Pre-osteoblasts were extracted from cranium of 1-week-old C57BL/6J and were cultured in DMEM containing 10% FBS and 1% penicillin and streptomycin. Mature osteoblasts were induced with 50 *μ*g/ml ascorbic acid and 10 mM *β*-glycerophosphate (Sigma-Aldrich, St. Louis, MO, USA), and the medium was changed every two days. Then, cells were stained with BCIP/NBT kit (CWBIO, Beijing, China) to detect ALP activity after 7 days. And 1% Alizarin red S (ARS) solution (pH 4.1) (Sigma-Aldrich) was applied to visualize calcium deposition in the extracellular matrix after 21 days. Mineralized calcium nodules were quantitatively assessed by measuring the stained extracts at 570 nm absorbance using a microplate reader (Bio-Tek Instruments, Winooski, VT, USA).

### 2.4. Bone Resorption

The bovine bone slices (Corning Inc., Corning, NY, USA) were placed beforehand in a 96-well plate, and then, BMMs were seeded on the bovine bone slices at a density of 8 × 10^3^ cells per well. Besides, we set up sham groups that seeded cells into the wells without bovine bone slices. After adding RANKL (50 ng/ml) and M-CSF (30 ng/ml) to promote mature osteoclasts generation for 5 days, the cells were treated with different concentrations of RR (0, 0.375, 0.75, and 1.5 *μ*M) for another 5 days. Finally, the bovine bone slices were taken out and brush off the remaining cells and then cleaned three times with PBS. The absorption degree on the bovine bone slices was observed by a Nikon scanning electron microscope (Nikon Corporation, Minato, Tokyo, Japan), and the data was quantitatively analyzed by Image J software (NIH, Bethesda, MD, USA).

### 2.5. Cytotoxicity Assay

The cell viability of RR on BMMs, osteoblasts (OBs), and BMSC was measured using the CCK-8 assay. The cells were cultured in 96-well plates (6 × 10^3^ cells/well) in triplicate overnight and then treated with indicated concentration of RR (0.195, 0.391, 0.781, 1.563, 3.125, 6.25, 12.5, 25, and 50 *μ*M) for 48 or 96 h. Afterward, all plates were changed with new medium and added 10 *μ*l CCK-8 buffer per well and then incubated at 5% CO_2_, 37°C for 1 h. The cell viability was detected using a microplate reader (Bio-Tek Instruments, Winooski, VT, USA) at absorbance of 450 nm wavelength.

### 2.6. RNA Extraction and Quantitative Real Time-PCR Assay

The cells were seeded (2 × 10^5^ cells/well) in 12-well plates and supplemented with 30 ng/ml MCSF, 50 ng/ml RANKL, and different concentrations of RR (0.375, 0.75, and 1.5 *μ*M) for 4 days. The cultured cells were washed three times with cold PBS and extracted total RNA with RNAiso Plus Kit (Takara Bio, Otsu, Japan) according to the instruction. The extracted RNA was then reverse-transcribed to obtain cDNA by conducting HiFiScript cDNA synthesis kit (CWBIO, Beijing, China). Quantitative real-time PCR was performed with an ABI Prism 7500 fast system (Applied Biosystems, Foster City, CA, USA) following specific cycling conditions: 95°C for 5 min, followed by 40 cycles at 95°C for 10 s and 60°C for 30 s, and a final step at 4°C for 10 min. The reaction was comprised of 5 *μ*l UltraSYBR Mixture (Takara Bio, Otsu, Japan), 1 *μ*l of cDNA, 3.6 *μ*l ddH_2_O, and 0.2 *μ*l each of forward and reverse primers (10 *μ*M). The primer sequences are shown in Table 1. The values of each target were calculated by the method of 2^−*ΔΔ*Ct^ and normalized to GAPDH.

### 2.7. Western Blotting Analysis

The BMMs were seeded into 6-well plates at a density of 5 × 10^5^ cells/well for indicated stimulation. Cultured cells were washed with cold PBS for three times. And then RIPA lysis buffer (Sigma-Aldrich, St. Louis, MO, USA)) with PMSF (1 mmol/L) or phosphatase inhibitor (CWBIO, Shanghai China) was added to each well to lyse the cells for 20 mins on ice. The supernatants were collected and dissolved in 1× loading buffer after centrifugation at 12,000*g* for 15 mins. Proteins were resolved on 10% SDS-PAGE gels and transferred to PVDF membranes (Millipore, Bedford, MA, USA). The membranes were blocked with quick blocking buffer at room temperature for 15 mins. Next, the protein bands were incubated with specific primary antibody (1 : 1,000 dilution) at 4°C overnight. After that, the protein bands, washed three times with TBST, were then incubated with the HRP-conjugated goat anti-mouse/rabbit IgG (1 : 2,000 dilution; Abcam) at room temperature (RT). The contents of protein on bands were visualized by using ECL western blotting reagents (Thermo Scientific Pierce, Rockford, IL, USA). Relative grey level of protein bands was measured by Image J software.

### 2.8. Immunofluorescence (IF) Staining and F-Actin Belt Staining

The BMMs were cultivated in a 96-well plate with the presence of RR. The cells washed with PBS three times and fixed in 4% paraformaldehyde for 15 mins at room temperature. Triton X-100 (0.1%, v/v) was carried out for 20 mins to permeabilize the cells. After blocking with goat serum, anti-NFATc1 antibody (1 : 200, Cell Signaling Technology, Danvers, MA, USA) was added to wells overnight at 4°C, followed by incubation with a goat anti-mouse Alexa Fluor-488-conjugated secondary antibody (Abcam) for an hour at RT. In order to visualize F-actin ring formation, rhodamine phalloidin was used for F-actin staining at room temperature away from light also for an hour. After removing excess dye by washing with PBS, DAPI (Beyotime Institute of Biotechnology, Shanghai, China) was utilized to stain nucleus for 15 mins at RT. Finally, the results were observed under a confocal microscope (NIKON A1Si, Nikon Corporation, Minato, Tokyo, Japan).

### 2.9. ROS Production Assay

Intracellular ROS levels were detected by ROS assay kit (Beyotime). Briefly, cells were seeded in six-well plate and pretreated with different conditions of RR for 24 hours with 50 ng/ml RANKL. Then, they were tested by a fluorescent probe DCFH-DA (1 : 1000 dissolved in a serum-free medium) and incubated 30 mins at 37°C. DCFH-DA freely passed through the cell membrane and was hydrolyzed to produce DCFH. Next, reactive oxygen species in cells can oxidize DCFH to generate fluorescent DCF. After incubation, the cells were washed with serum-free medium to remove excess dye. The fluorescence of DCF was measured using a confocal microscope (NIKON A1Si, Nikon Corporation, Minato, Tokyo, Japan), and the mean fluorescence intensity was quantitatively analyzed by Image J software.

### 2.10. Cell Transfection

The BMMs were cultured in *α*-MEM with 1% penicillin/streptomycin, 10% FBS, and 30 ng/ml M-CSF in an 37°C incubator with 5% CO_2_. The Raw 264.7 cells were cultured in RPMI 1640 Medium (Gibco, Gaithersburg, MD, USA) with 10% FBS. Before transfection, the BMMs were stimulated with 50 ng/ml RANKL for 4 hours and then transfected with MCU small-interfering RNA (siRNA), mouse MCU plasmids (NM_001033259.4), and negative control, which were purchased from Tsingke Biotechnology Co. (Beijing, China). After 6 hours, the cells were changed with fresh medium containing RANKL and indicated stimulations. Transfections were performed using TSnanofect transfection reagent (Tsingke Biotechnology Co., Beijing, China) according to the manufacturer's instructions. The si-RNA sequence used in this study is as follows: CAGAGACAGACAAUACUUATT.

### 2.11. Measurement of Calcium Concentration

According to manufacturer's instructions, a calcium colorimetric assay kit (Beyotime Biotechnology) was used to measure calcium concentration. Briefly, the Raw264.7 cells were cultivated in 6-well plate with RANKL and RR (1.5 *μ*M) stimulation for 24 or 48 hours and then washed with PBS and lysed with lysis buffer. Supernatants, collected after centrifugation, and working color solution were added, and then, the mixtures were incubated at RT for 10 mins to detect the absorbance at 575 nm through a microplate reader (MD Spectra Max i3x). Protein concentrations, used to normalize the amount of calcium, were measured through an BCA protein assay kit (Beyotime Biotechnology).

### 2.12. Ovariectomized (OVX)-Induced Bone Loss Mouse Model

All animal experiments were performed in accordance with the principles and procedures of the National Institutes of Health (NIH) Guide and the guidelines for the animal treatment of the first affiliated Hospital of Zhejiang University. The mice were anesthetized with 3 mg/ml pentobarbital and performed either bilateral ovariectomy (OVX) or a sham operation. We divided 25 healthy 8-week-old female C57BL/6J mice into 5 groups randomly (each; *n* = 5): Sham group (sham operation and injection with PBS), vehicle group (OVX and injection with PBS), alendronate sodium (AL) group (OVX and injection with 0.5 mg/kg AL) [2], low-dose group (OVX and injection with 2 mg/kg RR), and high-dose group (OVX and injection with 8 mg/kg RR). Four weeks after OVX, the treatment group was injected intraperitoneally with RR or alendronate sodium every other day for another 4 weeks to measure the therapeutic effects of RR. Besides, the mice were injected with calcein (12.5 mg/kg; Sigma) 10 days and 3 days before death. Uteri were isolated from mice and weighed to evaluate the effects of OVX at the end of 4 weeks. After sacrificing the experimental mouse, the right femurs of all groups were fixed in paraformaldehyde (PFA) for micro-CT as previous described [27], while the left femur and tibia of mice were fixed in 4% PFA and then decalcification for histological studies. The forelimbs of each mouse were kept in liquid nitrogen after dissection for the subsequent extraction of RNA and proteins.

### 2.13. Histological Analysis and Immunohistochemistry

The fixed left femur and tibia were immersed in 10% ethylenediaminetetraacetic acid (EDTA) for 4 weeks to decalcify and then embedded in paraffin to perform histological sections. The segments were examined by TRAP and H&E staining, using premium microscope known as Aperio Scanscope (Mt. Waverley, VIC, Australia) to observe and photograph. The number of TRAP-positive cells per field was calculated through Image-Pro Plus software. For immunohistochemistry (IHC), the sections of decalcified femur and tibia were incubated with anti-rabbit MCU antibody (1 : 500, Lot#ab272488, Abcam, USA) for 12 hours, followed by incubation with HRP-labeled secondary antibody for 50 mins at RT. The sections were visualized by Aperio Scanscope after staining with 3,3′-diaminobenzidine (Gene Tech, Shanghai, China) to assess the expression level of MCU protein. And the immunofluorescence of paraffin sections was performed as manufacturer's protocol described to analyze the location and level of MCU protein.

### 2.14. Calcein Double Fluorescent Labeling and von Kossa Staining

For calcein bone labeling, the mice were injected intraperitoneally with 12.5 mg/kg calcein (resolved in PBS) twice on the 10th day and 3rd day before sacrifice. The isolated right femurs of each group without decalcification were made into hard tissue slices. The average distance between the two fluorescent bands and the mineral apposition rate (MAR) was calculated by Image-Pro Plus software. For von Kossa staining, the undecalcified slices were flooded with a 2% silver nitrate solution and then exposed to UV lamp for 20 mins. Next, 5% sodium thiosulfate was used to treated for 2 mins. Finally, the slices were rapidly dehydrated. The staining results were observed using a Diaplan light microscope.

### 2.15. Statistical Analysis

Utilizing Prism 7 windows (GraphPad Software Inc., San Diego, CA, USA), all data were examined from triplicate experiments and stated as mean ± SEM. For statistical significance, one-way or two-way ANOVA and Student's *t* test were carried out. *P* < 0.05 was considered to be significant differences between groups.

## 3. Results

### 3.1. RR Inhibits Osteoclasts Formation and Bone Resorption In Vitro

The chemical structural formula of RR is shown in Figure 1(a). To further verify the cytotoxicity of the drug, we determined cell viability through CCK8 experiments for 48 and 96 hours to ensure that the concentration of the drug used in the article was within the safe range. As is shown in Figure 1(b), there was no cytotoxicity at the dose of 1.5 *μ*M. During RANKL-induced osteoclast formation, the addition of RR stimulation (0.375 *μ*M, 0.75 *μ*M, and 1.5 *μ*M) inhibited TRAP-positive multinuclear osteoclast formation in a dose-dependent manner (Figures 1(c) and 1(e)). At different time phase of osteoclast differentiation, the inhibitory effect of RR was found to be more significant at early stage (days 1-3) of osteoclast formation (Figures 1(d) and 1(f)). Moreover, F-actin rings that reflected the morphological changes of the mature osteoclasts were stained with phalloidin, and circumference of the F-actin ring was quantitatively analyzed (Figures 1(g) and 1(h)). The results showed that the formation of F-actin rings was significantly inhibited as the concentration of RR increased. In order to further verify the effect of RR on osteoclast function, bone resorption experiments found that RR inhibited bone resorption ability of dose dependently (Figures 1(i) and 1(j)). Based on the above results, it can be concluded that RR inhibits osteoclast formation and bone resorption in vitro without toxic effects on cells.

### 3.2. RR Inhibits Osteoclast-Specific Gene Expression

To verify the inhibitory effect of RR on the osteoclast formation, we investigated that RR inhibited the mRNA expression levels of bone-specific genes, including NFATc1, ACP5, DC-STAMP, CTR, CTSK, and ATP6v0d2 in a concentration dependent manner (Figure 2(a)). Moreover, the expression levels of ACP5, DC-STAMP, CTSK, and ATP6v0d2 were elevated under the stimulation of RANKL alone, while the expression of the above genes was downregulated after the addition of RR at the same time period (Figure 2(b)). Thus, RR downregulates the expression level of osteoclast-specific genes.

#### 3.2.1. RR Inhibits MCU Expression during Osteoclast Differentiation and Downregulates the Expression Level of NFATc1

To further explore the important role of RR during osteoclast formation, western blot results demonstrated that RR downregulated the RANKL-induced high expression of NFATc1 and c-Fos after stimulation of BMMs with 1.5 *μ*M RR for indicated different days. Besides, the MCU expression level also significantly reduced compared with the control group (Figures 3(a) and 3(b)). Similarly, with the addition of different concentrations of RR, the expression levels of NFATc1, c-Fos showed a gradual decrease as well (Figures 3(c) and 3(d)). As MCU acts as an intracellular calcium-channel protein that transported Ca^2+^ from cytoplasm to mitochondrial matrix, it can influence the intracellular calcium balance and even extracellular calcium entering the cells. The Ca^2+^ concentration was subsequently detected with stimulation of RANKL and RR. It was found that elevated intracellular calcium occurred within 24 hours of stimulation, while there was no difference after 48 h (Figure 3(e)). In terms of calcium in supernatant, calcium mobilized extracellularly increased at 48 hours of stimulation, which was consistent with declined intracellular calcium in all three experimental groups (Figure 3(f)). These results revealed that RR increased cytoplastic calcium levels for a short period of time, but did not affect osteoclasts calcium signaling directly. Additionally, being consistent with the results of western blot, immunofluorescence analysis manifested that RR stimulation attenuated the expression of NFATc1, which is a key transcription factor for activating osteoclast differentiation. And NFATc1 (marked with green fluorescence) hardly overlaps with the nucleus (marked with blue fluorescence) in the group of RR treatment, indicating that its nuclear translocation was hampered by RR (Figure 3(g)).

### 3.3. RR Inhibits MCU-Mediated ROS Production in Osteoclasts

According to previous literatures, RANKL promotes intracellular ROS production when inducing BMMs differentiation into osteoclasts, further activating the osteoclast differentiation signaling pathway and ultimately promoting osteoclast formation. As we can see in Figure 4(a), RANKL stimulate the production of total ROS using a fluorogenic dye (DCFDA), while RR significantly reduce the level of ROS in a dose-dependent manner. The fluorescence signal intensity was viewed under a fluorescence microscope, and the number of ROS-positive cells as well as the fluorescence intensity was quantified (Figures 4(b) and 4(c)). In addition, the mRNA levels of intracellular antioxidant enzymes, including catalase (CAT), heme oxygenase-1 (HMOX1), and glutathione reductase (Gsr), were upregulated. However, Kelch-like ECH-associated protein 1 (Keap1) dissociated from the nuclear factor-erythroid factor 2-related factor 2 (Nrf2) when the cells were subjected to oxidative stress. Nrf2 was activated to exert antioxidant stress, while Keap1 was gradually degraded, and its mRNA levels were gradually reduced (Figure 4(d)). Consistently, after transfection of Raw264.7 cells with small interfering RNA (si-RNA) to silence the MCU, it was found that the amount of ROS was significantly inhibited compared with the empty vector and the control group (Figures 4(e)–4(g)). Conversely, by transfecting Raw264.7 cells with plasmids to overexpress MCU, ROS production was obviously higher than that in the control group, whereas RR reinhibited ROS production after overexpression of MCU (Figures 4(h)–4(j)). In summary, we believe that MCU can promote RANKL-induced intracellular ROS production, and RR attenuated MCU-mediated ROS production by inhibiting MCU function and expression.

### 3.4. MCU Promotes RANKL-Induced Osteoclast Formation and Bone Resorption

To investigate the impact of MCU on osteoclasts differentiation, we have learned that RR is a potent inhibitor of MCU, blocking the entry of calcium from the cytoplasm into the mitochondrial matrix [28], thus affecting the internal environment of osteoclasts. So, we transfected osteoclasts with targeted si-RNA to knock down the expression of MCU, while an empty vector was used as a control. After osteoclasts induction with or without RANKL for 7 days, TRAP staining and quantitative statistics on the number and area of mature osteoclasts showed that MCU knockdown inhibited the differentiation of osteoclasts (Figures 5(a) and 5(b)). It was also indicated that after MCU knockdown, the expression levels of osteoclast-specific proteins NFATc1, c-Fos, ACP5, and CTSK were significantly declined (Figures 5(c) and 5(d)). In contrast, the overexpression of MCU in osteoclasts by plasmid transfection promoted osteoclast differentiation (Figures 5(e) and 5(f)) and the expression of osteoclast-specific proteins. These results further verified that MCU promote osteoclast differentiation and protein expression (Figures 5(g) and 5(h)). Moreover, the bone resorption experiments showed that MCU knockdown reduced the numbers of bone resorption pits, while MCU overexpression accelerated the osteoclast bone resorption capability (Figures 5(i) and 5(j)).

### 3.5. RR Inhibits Osteoclast Formation by Inhibiting the P38 MAPK Signaling Pathway via MCU

According to previous literature reports and experiments, the MAPKs family plays an important role in the process of osteoclast differentiation [29]. We analyzed the change in the phosphorylation level of pathway proteins using western blot with RR prestimulation. And the proteins were extracted after RANKL stimulation for 0, 15, 30, and 60 minutes. The results showed that the phosphorylated protein expression levels of p-P65, p-ERK, and p-JNK did not change significantly, while the phosphorylation level of P38 had the most significant inhibitory effect by RR at the 15 mins and 30 mins (Figures 6(a) and 6(b)). In order to further verify the relationship between p-P38, RR, and SB203580, an inhibitor of P38 MAPK signaling pathway acted simultaneously with RR on osteoclasts. The TRAP staining and quantitative analysis were performed after RANKL stimulation, which indicated that both RR and SB203580 inhibited osteoclast differentiation, and the inhibition effect was more significant under the combined action of the two (Figures 6(c) and 6(d)). Arachidonic acid (AA) has been shown to upregulate its expression levels as a P38 MAPK agonist [30]. As shown in Figure 6(e), the Raw264.7 cells are prestimulated with AA and RR, followed by the RANKL stimulation for indicated different times. Western blot results manifested that the rescue effect of P38-MAPK phosphorylation at the 15 mins was the most significant (Figure 6(f)). Similarly, AA had the same salvage effect on P38-MAPK phosphorylation levels at the 15 mins under the combined effect of RR and SB203580 (Figures 6(g) and 6(h)). To further verify the MCU on RR mediated P38 phosphorylation, the Raw264.7 was transfected with si-MCU and then treated with RANKL for 15 mins. The western blot results showed the efficiency of MCU silencing and the restrained phosphorylation level of P38 after MCU knockdown (Figures 6(i)–6(k)). In summary, RR inhibits osteoclast formation by inhibiting P38 phosphorylation and blocking downstream signaling pathways via MCU.

### 3.6. RR Promotes Osteogenesis Differentiation In Vitro

The above research results have proved that RR has a significant inhibitory effect on osteoclasts differentiation and function. In order to further explore the effect of RR on osteoblasts, we first determined the drug toxicity range of RR on primary osteoblasts through CCK8 experiments, and no cytotoxicity was observed at the concentration of 1.5 *μ*M (Figures 7(a) and 7(b)). Pre-osteoblasts were induced to differentiate by vitamin C and *β*-glycerosodium phosphate salts, and different concentrations of RR were added to assess the effects on osteoblasts differentiation. Alkaline phosphatase (ALP) is a signature enzyme for mature osteoblasts, and the ALP staining results showed that the osteogenesis was more remarkable compared with the undocumented group. Besides, the alizarin red S (ARS) staining, reflecting calcium precipitation, was promoted with RR stimulation for 21 days (Figures 7(c)–7(e)). The mRNA level of the MCU gradually decreased with the increased concentration of RR stimulation, resulting in increased intracellular calcium concentration in the meanwhile (Figures 7(f) and 7(g)). Calcium deposition in cellular may mostly contribute to osteoblasts differentiation. And, the gene levels of the osteoblast-specific genes ALP, Runx2, OPG, and OCN were also upregulated, which was consistent with the trend of MCU downregulated (Figures 7(h) and 7(i)). Similarly, with different concentrations of RR stimulated on BMSC for 7 days, the western blot results showed that the protein expression levels of Runx2, a key transcription factor for osteoblasts, and col1*α*, a differentiation-specific protein, increased significantly under the stimulation of RR (Figures 7(j) and 7(k)). Based on the above findings, we conclude that RR can promote the differentiation and function of pre-osteoblasts through MCU inhibition in vitro.

### 3.7. RR Plays a Vital Role in Alleviating against OVX-Induced Bone Loss In Vivo

This study explored the role of RR in vivo by constructing OVX-induced mouse animal models of osteoporosis and established the alendronate sodium (AL) treatment group as a positive control. The experimental mice are operated as shown in Figure 8(a). There was no influence found in the mice weight (Figure 8(b)). The protein and RNA were extracted from the isolated forelimbs of mice. The protein and mRNA expression level of the MCU in the OVX group were significantly increased compared with Sham group according to WB and qPCR analysis. After low-dose (2 mg/kg) and high-dose (8 mg/kg) RR treatment, protein and gene expression of the MCU were suppressed. However, in the AL-treated (0.5 mg/kg) positive control group, MCU expression was the highest (Figures 8(c)–8(e)) compared to all groups, and the reasons for this need to be further explored. After the treatment of AL and RR, the expression of osteoclast-specific genes CTSK and ATP6v0d2 was significantly downregulated compared with the vehicle group. The results of histo-immunofluorescence analysis also supported the distribution and expression level of MCU in various experimental groups (Figure 8(f)). The micro-CT study presented that significant bone loss arose in the OVX group, while RR-treated could ameliorate OVX-induced osteoporosis (Figure 8(g)). Histological analysis of the tibia and femur using H&E staining showed that RR reduced bone loss in mice (Figure 8(h)). More importantly, to determine the expression localization and the level of MCU in bone tissues, we used immunohistochemical staining results to observe that MCU was highly expressed in the cytoplasm of the vehicle group and AL-group and low expression in the Sham group and RR treatment group (Figure 8(i)). Furthermore, the remarkable decrease in the TRAP-positive cell numbers by RR was obviously revealed from TRAP staining of femurs, proving that RR inhibited osteoclast formation in vivo (Figure 8(j)). To further explore the consequences of osteoblast with RR treatment, von Kossa staining and calcein double fluorescent labeling were examined for femoral mineralization area and deposition rate. In the OVX-induced osteoporosis mice model, the von Kossa staining of femurs displayed that the ratio of mineralized area to bone surface area (MS/BS %) and the density of the trabecular were decreased, while RR treatment can partly reverse these results. Besides, the MAR of the femur, showed by calcein double fluorescent labeling, was significantly improved by RR when compared with the vehicle group (Figures 8(k) and 8(l)). As confirmed by the above results, RR reduced bone mass loss in OVX mice by inhibiting the expression of MCU.

## 4. Discussion

Bone tissue is constantly reshaped throughout a person's life. Aging, decreased estrogen levels during menopause in women, and oxidative stress are common triggers for osteoporosis. The underlying cause of osteoporosis is an imbalance between osteoclast-mediated bone resorption and osteoblast-mediated bone formation [31]. In recent years, there have been diversities of drugs and targets for the treatment of osteoporosis, such as estrogen replacement therapy and drugs like dihydric phosphate, whereas the side effects of drugs, including vaginal bleeding, deep vein embolism [32], breast cancer [33], and necrosis of the mandible [34], limited their clinical use. Therefore, finding a new therapeutic target and its corresponding inhibitory drugs can provide a new direction for the treatment of osteoporosis. In this study, we demonstrated for the first time that MCU play an important part in bone metabolism. The MCU inhibitor RR was able to inhibit osteoclast differentiation and bone resorption by attenuating ROS production and P38 MAPK phosphorylation levels, while also promoting osteogenesis and treating OVX mice in vivo (Figure 9).

Our team has summarized the close relationship between MCU and ROS production and elaborated the influence of MCU on cellular energy metabolism and cell death in a review published earlier. The MCU acts as an intracellular calcium-channel protein that maintains the homeostatic balance of calcium between the cytoplasm and mitochondrial matrix [35]. Calcium is an important factor in bone mineralization, and the loss of calcium ions in osteoclasts leads to changes in their morphology and function, thereby inhibiting osteoclast activity [36]. RR is able to enter the cell and bind directly to the MCU on the mitochondria, blocking calcium channels [26], and the changes in intracellular ions lead to inhibition of osteoclast function. Therefore, the biological activity of RR was first verified in the experiment. We observed that the differentiation and the F-actin rings formation of osteoclasts were inhibited by RR within the toxicity range of the drug dose. At the same time, the bovine bone slices experiment also proved that RR inhibited the bone resorption function of osteoclasts. These results demonstrate the inhibitory effect of RR on osteoclast differentiation and function.

To further explore how RR affects osteoclasts and osteoblasts through MCU, we have conducted experimental verification of the relationship between MCU and ROS. Previous studies have reported that RANKL can induce increased ROS production within osteoclasts, and ROS can activate the downstream of P38 MAPK signaling pathway and promote osteoclast formation [37]. Furthermore, studies have shown that inflammatory response stimulation and oxidative stress lead to increased ROS production and induction of osteoblast apoptosis [38]. In our research, RANKL-induced increasing ROS production causes cells under oxidative stress, leading to upregulation of antioxidant enzyme expression and activity. The Nrf2/Keap1/antioxidant-responsive element (ARE) pathway is an important factor in regulating antioxidant enzyme gene expression [39]. When the oxidizing ions bind to the Keap1 protein, it causes the dissociation of Nrf2 from Keap1 within the cytoplasm. Dissociated Keap1 is degraded by the proteasome, while Nrf2 enters into nuclear to activate the ARE, which is located in the transcription promoter region. Activated ARE exerts the major antioxidant effects in cells by promoting the expression of CAT, HMOX1, Gsr, and other enzymes that play a major antioxidant role [40]. In this study, we demonstrated that RR is able to decline the production of ROS via overexpressing or silencing MCU. And the qPCR results also showed that the expression of antioxidant enzymes in osteoclasts was significantly upregulated with the RR-treated. Meanwhile, osteogenesis-specific staining, qPCR, and WB results all show that RR has a promoting effect on osteoblast formation and differentiation. However, whether the specific mechanism is related to ROS still needs to be further explored.

The signaling pathways of osteoclastogenesis have formed a complex network with the diversities of explorations and researches. The NF-*κ*B and MAPK protein family are two important signaling pathways for osteoclast formation. The MAPK family, including ERKs, JNKs, and P38, is phosphorylated under RANKL stimulation and is involved in osteoclast differentiation [41]. The results of WB in the experiment proved that RR inhibited phosphorylation level of P38, but did not have an effect on ERKs, JNKs, and NF-*κ*B signaling pathways. At the same time, under the addition of the P38 agonist AA and the inhibitor SB203580, the inhibition effect of RR on the P38 MAPK signaling pathway was indeed verified. Numerous studies have demonstrated that NFATc1 is a key transcription factor for osteoclast differentiation and is capable of continuous self-amplification [42, 43]. NFATc1 knockout mice exhibit severely impaired osteoclast formation and significantly suppressed transcription of osteoclast-specific genes [6]. Our findings confirm that the mRNA and protein expression levels of RANKL-induced NFATc1 are inhibited by RR and that the nuclear localization of NFATc1 is also affected by RR. Consistently, the mRNA expression levels of the osteoclast-specific genes, such as ACP5, DC-STAMP, CTR, CTSK, and ATP6v0d2, which is directly regulated by NFATc1, were also suppressed. It is reported that intracellular calcium oscillations are also closely related to NFATc1. Under physiological conditions, RANKL stimulates the release of calcium within cytoplasm in osteoclasts, and then, calcium oscillations trigger an increase in NFATc1 activity as well as self-amplification [44]. In this study, MCU overexpression can promote the increase in the expression of NFATc1. In contrast, when the MCU expression is knocked down, the expression of NFATc1 is reduced. RR prevents the entry of calcium ions from the cytoplasm into the mitochondrial matrix by inhibiting the MCU. The instantaneous increase of intracellular calcium may enhance the activity of NFATc1, but the sustained high intracellular calcium concentration blocks the energy metabolism in the cells and prevents calcium influx from outside [45–47], causing NFATc1 dysfunction, which may be one of the important mechanisms of RR affecting bone formation. Recent studies have found that other compounds also alleviate the osteoclastogenesis and ovariectomy-induced osteoporosis via suppressing RANKL-induced ROS production and NFATc1 activation. In the researches of Chen et al. [48] and Liu et al. [49], they also found that Pseurotin A and Loureirin B can inhibit ROS production and NFATc1 activation. However, the mechanism by which the compound mediates reactive oxygen species production has not been directly verified. MCU plays an important role in energy metabolism and various enzyme activities by mediating cellular calcium balance. The dehydrogenases that participate in tricarboxylic acid cycle and even the conductance of complexes I, III, IV, and V in oxidative phosphorylation are sensitive to mitochondrial Ca^2+^, which is reported to be the main source of ROS [50]. In addition, the relationship between MCU and bone metabolism has rarely been investigated. Consequently, RR is worthy of study in that it can inhibit MCU expression and function to influence bone metabolism.

Based on the above experimental results in vitro, we verified the potential therapeutic effect of RR in vivo by constructing a mouse model of OVX-induced osteoporosis. WB, immunofluorescence staining, and immunohistochemical analysis showed that RR inhibited MCU expression in vivo. According to the results of TRAP staining and H&E staining, RR can have a therapeutic effect on bone mass loss to treat osteoporosis. The expression of osteoclast-specific genes CTSK and ATP6v0d2 was significantly reduced in the RR treatment group, which was consistent with the results of experiments in vitro. Moreover, von Kossa staining and calcein double fluorescent labeling displayed that RR can promote boss formation in vivo to reverse osteoporosis. As a positive control, the AL group had a significant therapeutic effect on osteoporosis, but the expression of MCU showed an abnormal increase. As a third-generation diphosphonate, alendronate sodium affects intracellular calcium concentration by inhibiting ATP-dependent enzymes related to osteoclast function, altering cytoskeleton and morphology. Alendronate sodium is able to free up from the bone to augment the leakage of calcium from osteoclasts, reducing calcium levels in the cytoplasm [51, 52]. We hypothesized that AL may promote calcium elimination within the cytoplasm by increasing MCU that facilitates calcium entering into mitochondria, and the specific mechanism still needs to be further explored.

## 5. Conclusion

In conclusion, our study demonstrated for the first time that the MCU inhibitor RR was able to inhibit osteoclast formation and bone resorption by inhibiting ROS, P38 MAPK, and NFATc1 and validated its potential therapeutic effects in osteoporosis animal models. Moreover, it was also found that the drug also has a positive effect on osteogenesis. Therefore, RR can inhibit bone mass loss and promote osteogenesis, thus having a therapeutic effect on osteoporosis, which opens up a new therapeutic target for the study of bone metabolic diseases.

## Figures and Tables

**Figure 1:** RR inhibits RANKL-induced osteoclast formation in vitro. (a) The chemical structural formula of RR; (b) The cell viability of different concentration gradients RR-stimulated BMMs after 48 h and 96 h. (c) BMMs were induced by RANKL with 25 ng/ml M-CSF and 50 ng/ml and stimulated with RR at different concentrations (0.375 *μ*M, 0.75 *μ*M, and 1.5 *μ*M) for 7 days. Osteoclast formation results were shown using TRAP staining, scale bar = 100 *μ*m. (d) BMMs were induced with 25 ng/ml M-CSF and 50 ng/ml RANKL for a total of 7 days, and 1.5 *μ*M RR was added at indicated periods of induction. TRAP staining results were shown, scale bar = 100 *μ*m. (e, f) Quantitative results of multinuclear TRAP-positive cell numbers and the area occupied. (g) The BMMs were planted in a 96-well plate with approximately 8 × 10^3^ cells per well and stimulated with 25 ng/ml M-CSF and 50 ng/ml RANKL for 5 days while adding the different concentrations of RR described above. The cells were fixed with PFA and after 1% Triton 100× membrane breakdown. F-actin ring was stained with phalloidin, scale bar = 100 *μ*m. (h) Quantitative analysis of the circumference of the F-actin ring using Image J software. (i) Representative image of osteoclast bone absorption pits, scale bar = 500 *μ*m. (j) Quantification of bone absorption pits in different groups. Data was presented as means ± SEM; *n* = 3; ^∗^*p* < 0.05, ^∗∗^*p* < 0.01, ^∗∗∗^*p* < 0.001, ^∗∗∗∗^*p* < 0.0001.

**Figure 2:** RR inhibits osteoclast-specific genes expression levels. (a) The Raw264.7 cells were stimulated with M-CSF and RANKL for 5 days, while adding indicated different concentrations of RR, the mRNA expression levels of osteoclast-specific genes, including NFATc1, ACP5, DC-STAMP, CTR, ATP6v0d2, and CTSK, were detected by qPCR, and normalized relative to GAPDH. (b) Raw264.7 cells were stimulated with M-CSF and RANKL for 5 days, and 1.5 *μ*M RR was added at the same time for 1 d, 3 d, and 5 d, respectively, and the osteoclast specific gene expression level was detected by qPCR. Data was presented as means ± SEM; *n* = 3; ^∗^*p* < 0.05, ^∗∗^*p* < 0.01, ^∗∗∗^*p* < 0.001, ^∗∗∗∗^*p* < 0.0001.

**Figure 3:** RR inhibits the MCU expression and downregulates the expression of NFATc1. (a) The BMMs were planted in a 6-well plate, M-CSF and RANKL stimulation were added, and 1.5 *μ*M RR was added to stimulate 0 d, 3 d, 5 d, and 7 d, respectively. Western blot was used to show protein expression levels of NFATc1, c-Fos, and MCU. (b) Image J was used to quantitatively detect the expression of NFATc1, c-Fos, and MCU, normalized relatively to GAPDH. (c) After adding M-CSF, RANKL, and different concentrations of RR to stimulate BMM for 7 days, protein expression levels of NFATc1 and c-Fos were displayed by western blot. (d) Quantitative analysis of protein expression levels of NFATc1 and c-Fos, normalized relatively to GAPDH. (e) The RAW264.7 cells were treated with or without RANKL and RR for 24 h and 48 h, and then, intracellular calcium concentration was measured. Normalized relatively to protein concentrations per well. (f) The calcium concentration in supernatant of RAW264.7 cells, normalized to protein concentrations. (g) BMM cells were stimulated with RANKL in the presence or absence of RR (1.5 *μ*M), and the expression and localization of NFATc1 were analyzed using immunofluorescence. Scale bar = 100 *μ*m. Data was presented as means ± SEM; *n* = 3; ^∗^*p* < 0.05, ^∗∗^*p* < 0.01, ^∗∗∗^*p* < 0.001, ^∗∗∗∗^*p* < 0.0001.

**Figure 4:** RR suppresses MCU-dependent ROS generation. (a) Raw264.7 cells were planted in a 6-well plate, with or without RANKL and different concentrations of RR stimulation, using DCFH-DA probes to show RANKL-induced ROS production, scale bar = 100 *μ*m. (b) Quantitative analysis of ROS positive cell number by Image J software. (c) Quantitative analysis of DCF relative fluorescence intensity in cells per well. (d) Raw264.7 cells were stimulated with RANKL and different concentrations of RR, and intracellular antioxidant enzyme mRNA levels were shown using qPCR results. (e) With si-MCU or empty vector transfection into Raw264.7 cells with the addition of RANKL stimulation, DCFH-DA probe showed RANKL-induced ROS production, scale bar = 100 *μ*m. (f) Quantitative analysis of ROS positive cell numbers. (g) Quantitative analysis results of DCF relative fluorescence intensity in cells per well. (h) Raw264.7 cells were transfected with MCU plasmids or empty vectors with the addition of RANKL stimulation, and DCFH-DA probe showed total ROS production, scale bar = 100 *μ*m. (i) Quantification of ROS positive cell numbers. (j) Quantitative analysis of DCF relative fluorescence intensity in cells per well. BF: bright field; DCFH-DA: 2',7'-dichlorofluorescin diacetate; Data was presented as means ± SEM; *n* = 3; ^∗^*p* < 0.05, ^∗∗^*p* < 0.01, ^∗∗∗^*p* < 0.001, ^∗∗∗∗^*p* < 0.0001.

**Figure 5:** MCU promotes osteoclast differentiation and absorption function. (a) The BMMs were planted in 96-well plates with a cell count of about 8 × 10^3^/well, si-MCU, or empty vector and were transfected into BMMs, adding M-CSF in the presence or absence of RANKL to induce osteoclast differentiation for 5 days. TRAP staining was utilized to show differentiation results. (b) Quantification of the TRAP-positive multinuclear cell numbers and the area occupied by image J software. (c) si-MCU or empty vector is transfected into Raw264.7 cells, and osteoclast-specific proteins and transfection efficiency of MCU silencing were showed by western blot after RANKL stimulation for 48 h. (d) Image J was used to quantitatively detect the gray value of the protein bands, normalized to *β*-actin (e) TRAP staining results after transfecting MCU plasmid or empty vector into the BMMs and adding RANKL and M-CSF to induce differentiation for 5 days. (f) Quantitative results of the TRAP-positive multinuclear cell numbers and the area occupied. (g) The Raw264.7 cells were transfected MCU plasmid or empty vector and stimulated with RANKL for 48 hours, and western blot was used to display osteoclast-specific proteins and transfection efficiency of MCU overexpression. (h) Image J was used to quantitatively detect the gray value of the protein band, normalized to GAPDH. (i) The bone slices were placed in a 96-well plate before planting BMMs. The cells were transfected with MCU plasmid and si-MCU and treated with RANKL to induce osteoclast. Bone resorption pits on bone slices under electron microscopy scanning. (j) Quantitative results of bone resorption pits, scale bar = 500 *μ*m. Data was presented as means ± SEM; *n* = 3; ^∗^*p* < 0.05, ^∗∗^*p* < 0.01, ^∗∗∗∗^*p* < 0.0001.

**Figure 6:** RR inhibits the osteoclast P38 MAPK signaling pathway via MCU. (a) Raw264.7 cells were planted in a 6-well plate until the cell confluency reaches 90%, treated with serum-free medium starvation for 2 h, and then replaced with serum-containing medium, and pretreated with or without RR (1.5 *μ*M) for 2 h before stimulation with RANKL for 0, 15, 30, and 60 min. The cells were lysed with RIPA, and the expression of p-P65, P65, p-ERK, ERK, p-JNK, JNK, p-P38, and P38 was displayed with western blot. (b) Quantitative analysis results of p-P65, p-ERK, p-JNK, and p-P38 relative to P65, ERK, JNK, and P38 ratios are displayed. (c) BMMs were planted in 96-well plates, with the addition of RANKL, SB203580 (10 *μ*M), and RR (1.5 *μ*M) for 5 days, and osteoclast differentiation results were shown by TRAP staining. (d) Quantitative results of TRAP-positive multinuclear cells and area occupied. (e) Raw264.7 cells were planted in a 6-well plate, treated with serum-free medium starvation for 2 h, and then replaced with serum-containing medium and pretreated with or without RR (1.5 *μ*M) and AA (10 *μ*M) for 2 h before stimulation with RANKL for 0, 15, and 30 min. Western blot showed the expression of p-P38 and P38. (f) Quantitative analysis of the p-P38 relative to P38 ratio at different stimulus times. (g) The Raw264.7 cells were starved with serum-free medium for 2 h, and then replaced with serum-containing medium with or without RR (1.5 *μ*M), AA (10 *μ*M), and SB203580 (10 *μ*M) for 2 h, and then stimulated with RANKL for 15 min. Western blot was used to show the expression of p-P38 and P38 expression. (h) Quantitative analysis of the p-P38 relative to P38 ratio. (i) The Raw264.7 were pre-transfected with si-MCU for 6 h, and then, the proteins were extracted after different times of RANKL stimulation. The western blot results showed the expression of p-P38, P38, and MCU. (j–k) Quantification of protein band gray values by Image J statistics. The data was presented as means ± SEM; *n* = 3; ^∗^*p* < 0.05, ^∗∗^*p* < 0.01, ^∗∗∗∗^*p* < 0.0001, normalized to *β*-actin.

**Figure 7:** RR promotes osteoblast differentiation as well as osteogenesis gene expression. (a–b) Cell viability of pre-osteoblasts with RR-treated for 48 h and 96 h. (c) After stimulating primary osteoblasts with osteogenesis induction solution (50 *μ*g/ml vitamin C, 10 mM *β*-glycerol) and different concentrations of RR for 7 and 21 days. Representative image of ALP staining and ARS staining to show osteogenesis differentiation results. (d) ALP activity was detected at different concentrations of RR after stimulating primary osteoblasts for 7 days. (e) Different concentrations of RR stimulated pre-osteoblasts for 21 days. After using ARS staining, calcium nodules were dissolved, and the absorbance value of the lysate solution at 570 nm was determined. (f) Pre-osteoblasts were stimulated with the indicated different concentrations of RR for 7 days, using qPCR to show the mRNA level of the MCU. (g) Primary osteoblasts treated with or without osteogenic induction (OI) and RR (0.75 *μ*M) for 48 h, and then, intracellular calcium concentration was measured. (h) The mRNA level of OPG, OCN, and OSX with MCU knockdown or not. (i) The relative mRNA expression level of osteoblast-specific genes, including ALP, Runx2, OPG, and OCN. (j) The bone-forming induction solution and different concentrations of RR (0.375 *μ*M, 0.75 *μ*M, and 1.5 *μ*M) were used to stimulate BMSCs for 7 days, and the western blot results showed the protein expression levels of Runx2 and Col1*α*. (k) Quantitative analysis of protein expression levels, normalized to GAPDH. Data was presented as means ± SEM; *n* = 3; ^∗^*p* < 0.05, ^∗∗^*p* < 0.01, ^∗∗∗^*p* < 0.001, ^∗∗∗∗^*p* < 0.0001.

**Figure 8:** RR plays a vital role in alleviating against OVX-induced bone loss in vivo. (a) Representative image of experimental mouse operation processing mode. (b) Weight change diagram of C57BL/6J mice before and after OVX surgery. (c) Mice forelimb bone tissue was isolated of from each experimental group. Adding tissue lysate to extract tissue protein, MCU-specific primary antibody was used to show the results by western blot. (d) Quantitative analysis of protein expression, normalized to *β*-actin. (e) Tissue total RNA was extracted from mice forelimb, and the mRNA expression levels of CTSK and ATP6v0d2 were displayed by qPCR. (f) Immunofluorescence staining to detect the expression of the MCU, scale bar = 500 *μ*m. (g) Representative micro-CT images of 3D demonstrating that OVX-induced osteoporosis was prevented by RR treatment. (h) H&E staining results detect bone mass loss, scale bar = 100 *μ*m. (i) Immunohistochemical staining shows MCU expression and distribution, scale bar = 50 *μ*m. (j) Representative image of TRAP staining and the TRAP positive osteoclast numbers per field of every specimen were examined, scale bar = 20 *μ*m. (k) The von Kossa staining of femurs was used for the measurement of MS/BS (%), scale bar = 100 *μ*m. (l) Calcein double fluorescent labeling to detect the femur mineral apposition rate (MAR) in mice, scale bar = 20 *μ*m. Data was presented as means ± SEM; *n* = 3; ^∗^*p* < 0.05, ^∗∗^*p* < 0.01, ^∗∗∗∗^*p* < 0.0001.

**Figure 9:** A schematic diagram for the mechanism of RR on osteoblast and osteoclast. RANKL is supposed to stimulate the BMMs to produce ROS and activate the downstream P38 MAPK signaling pathway to promote NFATc1 upregulation and mature osteoclast formation. By binding to the MCU on the intermembrane of mitochondria, RR inhibits MCU function and its expression to reduce ROS production. Besides, the phosphorylation of P38 and the activation of downstream signaling pathways are also inhibited, resulting in the disruption of mature osteoclasts differentiation. Meanwhile, the osteoblastogenesis is also facilitated under the treatment of RR.

**Table 1:** Mice primer pair sequences.

Genes	Forward (5′-3′)	Reverse (5′-3′)
MCU	AAAGGAGCCAAAAAGTCACG	AACGGCGTGAGTTACAAACA
HMOX1	GGCTTTAAGCTGGTGATGGCT	GGCGTGCAAGGGATGATTTC
SOD	CACTTCGAGCAGAAGGCAAG	CCCCATACTGATGGACGTGG
CAT	AAGATTGCCTTCTCCGGGTG	GACATCAGGTCTCTGCGAGG
Gsr	TGGCACTTGCGTGAATGTTG	TGTTCAGGCGGCTCACATAG
Keap1	TGCCCCTGTGGTCAAAGTG	GGTTCGGTTACCGTCCTGC
CTSK	CTTCCAATACGTGCAGCAGA	TCTTCAGGGCTTTCTCGTTC
Trap	CTGGAGTGCACGATGCCAGCGACA	TCCGTGCTCGGCGATGGACCAGA
c − Fos	CCAGTCAAGAGCATCAGCAA	AAGTAGTGCAGCCCGGAGTA
NFATc1	CCGTTGCTTCCAAAAATAACA	TGTGGGATGTGAACTCGGAA
Atp6v0d2	GACCCTGTGGCACTTTTTGTATTC	GCTTGCATTTGGGGAATCTATC
DC − STAMP	AAAACCCTTGGGCTGTTCTT	AATCATGGACGACTCCTTGG
ALP	CCAACTCTTTTGTGCCAGAGA	GGCTACATTGGTGTTGAGCTTTT
OCN	GAGGGCAATAAGGTAGTGAACAGA	AAGCCATACTGGTTTGATAGCTCG
Runx2	TTCTCCAACCCACGAATGCAC	CAGGTACGTGTGGTAGTGAGT
OPG	ACCCAGAAGACTGTGGATGG	CACATTGGGGGTAGGAACAC
GAPDH	GCACAGTCAAGGCCGAGAAT	GCCTTCTCCATGGTGGTGAA 3

## Data Availability

Data generated from this work and presented in this manuscript is available upon request from the corresponding author.
